The article "Observation of the Curative Effect of Acupuncture for Tonifying Kidney and Removing Blood Stasis Combined with Radiofrequency Surgery in Patients with NSCLC and the Diagnostic Efficacy of Combined Detection of NTx, BGP, and CYFRA21-1 in the Occurrence of Bone Metastases" was retracted in 2023. Reasons: signs of a paper mill; suspected computer-generated content; unreliable results or conclusions; lack of ethics approval or compliance.

# Observation of the Curative Effect of Acupuncture for Tonifying Kidney and Removing Blood Stasis Combined with Radiofrequency Surgery in Patients with NSCLC and the Diagnostic Efficacy of Combined Detection of NTx, BGP, and CYFRA21-1 in the Occurrence of Bone Metastases

**DOI:** 10.1155/2022/8157157

**Published:** 2022-09-28

**Authors:** Ge Song, Tian Jiang, Ying Wang, Tao Gu, Wentao Li

**Affiliations:** ^1^Deparment of Interventional Radiology, Fudan University Shanghai Cancer Center, Shanghai 200032, China; ^2^Institute of Traditional Chinese Medicine, Nantong Liangchun Hospital of Traditional Chinese Medicine, Nantong 226009, China

## Abstract

The curative effect observation of acupuncture for tonifying kidney and removing blood stasis combined with radiofrequency surgery in patients with non-small-cell lung carcinoma (NSCLC) and the diagnostic efficacy of combined detection of NTx, BGP, and CYFRA21-1 for bone metastases are investigated. 122 NSCLC patients admitted to our hospital from January 2019 to December 2021 are selected for the examination, and the two sets of patients are randomly divided into the study set and the control set using the random number table method, with 61 cases in each set. Patients in the control set are given CT-guided percutaneous radiofrequency ablation therapy, and patients in the study set are given a combination of acupuncture therapy for tonifying the kidney and removing blood stasis on the basis of the therapy of the control set. The experimental results show that for NSCLC patients, the application of kidney-tonifying and stasis-removing acupuncture therapy combined with radiofrequency surgery can notoriously enhance the clinical therapy effect and enhance the quality of life of patients, and the detection of NTx, BGP, and CYFRA21-1 indicators can effectively predict the prognosis.

## 1. Introduction

Lung carcinoma is one of the most common carcinomas that seriously affect the safety of human life. Non-small-cell lung carcinoma (NSCLC) accounts for a relatively high proportion of lung carcinoma. With the acceleration of aging process, its morbidity and mortality are increasing. Most patients are already in the middle and late stage when diagnosed, which affects the prognosis and makes it difficult to carry out radical surgery [1]. Therefore, effective therapies need to be explored to enhance patients' lives [2]. Percutaneous radiofrequency ablation is a new minimally invasive technique, which combined with radiotherapy and chemotherapy, opens up a new approach for clinical therapy of tumors [3]. However, it does not relieve patients' pain well. The World Health Organization suggests that opioids can be used to relieve moderate to severe carcinoma pain, but due to a variety of factors such as side effects and high cost of drugs, there are still a large number of patients with unsatisfactory pain relief effect due to other reasons [4, 5].

The article "Observation of the Curative Effect of Acupuncture for Tonifying Kidney and Removing Blood Stasis Combined with Radiofrequency Surgery in Patients with NSCLC and the Diagnostic Efficacy of Combined Detection of NTx, BGP, and CYFRA21-1 in the Occurrence of Bone Metastases" was retracted in 2023. Reasons: signs of a paper mill; suspected computer-generated content; unreliable results or conclusions; lack of ethics approval or compliance.

In recent years, TCM Bushen Quyu acupuncture has an extensive therapeutic effect on carcinoma patients, which can promote qi and blood circulation, warm yang and clear collatals, and relieve pain [6, 7]. However, currently there is no relevant examination on the efficacy of kidney-tonifying and stasis-removing acupuncture combined with radiofrequency therapy on NSCLC patients. To sum up, this examination included NSCLC patients treated in our hospital and applied kidney-tonifying and stasis-removing acupuncture combined with radiofrequency therapy to analyze its clinical efficacy, aiming to provide reference for the later clinical therapy of NSCLC.

The rest of this paper is organized as follows: Section 2 discusses related work, followed by clinical data and the proposed treatment method designed in Section 3.  Section 4 shows the experimental results, and Section 5 briefly summarizes the whole text, and points out the future research directions.

## 2. Related Work

NSCLC is one of the most common malignant tumors in the clinic, and its morbidity and mortality are high. Most of the patients are in the middle and advanced stages of diagnosis, losing the opportunity for surgery, and the clinical therapy is difficult [8]. Today, chemotherapy in modern remedy is often used to treat non-small-cell lung carcinoma, but it has many toxic and side effects, such as gastrointestinal reactions, bone marrow suppression, and subjoined performance status, which reduces patient compliance and leads to a poor prognosis [9]. Studies have found that the combination of traditional Chinese and Western remedy in the therapy of this ailment can complement each other's strengths. This examination found that the total effective rate in the study set was 90.16%, which was notoriously higher than 67.21% in the control set; after therapy, the KPS scores of the two sets were notoriously increased, and the NRS scores were subjoined, and the KPS score of the study set was notoriously higher than that of the control set. In the control set, the NRS score of the study set was notoriously lower than that of the control set (*p* < 0.05), because the TCM external therapy plays an important role in the therapy of pain, rich experience and theory have been accumulated [10]. “Lingshu” emphasizes “Meridians are interested in life and death, cure all ailments, and correct deficiency and excess.” It points out that acupuncture points can regulate qi and blood, dredge the meridians and then achieve pain relief, make acupuncture feel “qi to the ailment area,” regulate the functions of the viscera, and enhance qi blood dysfunction to achieve the purpose of reconciling qi and blood, from the effect of removing blood stasis and relieving pain [11]. Xuanzhong acupoint is the gathering place of the qi meridian Shaoyang foot and is also the essence of the eight associations, while Taixi needle is the infusion point and origin of the kidney meridian of Shaoyin foot, which has the functions of invigorating the kidney, strengthening the kidney, and promoting the qi of the kidney. At the same time, acupuncture can achieve the effects of invigorating the kidney, regulating qi, and relieving pain. Xuehai acupoint is one of the key points of the spleen meridian and Taiyin. The Yellow Emperor's Classic of Internal Medicine emphasizes that acupuncture and moxibustion focus on “healing the heart” [12]. Lung carcinoma patients with bone metastases have been affected and tortured by carcinoma pain for a long time and are prone to pessimism, disappointment, anxiety, depression, and other emotions. The psychological pressure is large, and the tolerance to pain is further reduced. Acupuncture and moxibustion can guide patients to concentrate, maintaining a calm state of mind is conducive to the conduction of meridian qi, and the patient's own thoughts are used to make the qi go to the sick place and relieve pain [13].

90% of bone is composed of collagen. When osteolytic lesions occur, the enhanced activity of osteoclasts leads to the degradation of collagen fibers to produce metabolites such as NTx, which enter the circulatory system and are finally excreted from the kidneys. NTx is currently considered to be a relatively sensitive marker of osteolytic bone metabolism [14]. Zhang and Lv [15] found that the regression decomposition was used to evaluate the correlation between the standard of NTx and the diagnosis of osteolytic lesions in patients with malignant tumors, and found that NTx has a good diagnostic value for bone metastasis of malignant tumors. In this examination, after therapy, the standards of NTx, BGP, and CYFRA21-1 in the two sets were enhanced, and the enhancement effect in the study set was notoriously better than that in the control set (all *p* < 0.05); the incidence of bone metastases in the study set was 14.75%, notoriously the bone metastasis rate was 49.18% lower than that in the control set (*p* < 0.05); the standards of NTx, BGP, and CYFRA21-1 in the bone metastasis set were notoriously higher than those in the nonbone metastasis set (all *p* < 0.05); and Ci [16] scholar. The reported sensitivity of NTx in diagnosing bone metastasis is 87.2%, and the specificity is 86.7%, which is relatively higher than the diagnosis results in this paper. The decomposition suggests that the examination by Chen et al. is different, while NTx may be affected by a high-fat diet. The specific binding protein BGP is released during bone formation and resorption. Conticchio et al. [17] studied the value of serum BGP standards in the diagnosis of lung carcinoma bone metastasis and found that the serum BGP standards were comparable between lung carcinoma patients and healthy people and between lung carcinoma patients with different pathological types, while the serum BGP standards in lung carcinoma patients with bone metastases were notoriously higher than the normal humans and patients without bone metastases. Cytokeratin 19 is mainly distributed in the lung tissue, especially in the cytoplasm of lung tumor epithelial cells. When alveolar epithelial cells undergo apoptosis, it can be degraded into soluble substances under the action of activated proteases, and then released into the blood circulation, resulting in serum CYFRA21-1 standards increased [18]. As an important chemical marker of the tumor immune tissue, CYFRA21-1 has a high reference significance for the clinical diagnosis, ailment judgment, and efficacy evaluation of non-small-cell lung carcinoma. Therefore, the early application of tumor suppressor drugs to treat non-small-cell lung carcinoma can prevent the formation of drug resistance. It can maximize the effect of killing tumor cells and enhance the therapeutic effect [19].

The article "Observation of the Curative Effect of Acupuncture for Tonifying Kidney and Removing Blood Stasis Combined with Radiofrequency Surgery in Patients with NSCLC and the Diagnostic Efficacy of Combined Detection of NTx, BGP, and CYFRA21-1 in the Occurrence of Bone Metastases" was retracted in 2023. Reasons: signs of a paper mill; suspected computer-generated content; unreliable results or conclusions; lack of ethics approval or compliance.

## 3. Clinical Data and the Proposed Treatment Method

### 3.1. Clinical Data

In this examination, 122 NSCLC patients admitted to our hospital from January 2019 to December 2021 are selected to carry out the examination. The two sets of patients are randomly divided into the study set and control set using the random number table method, with 61 patients in each set. There are 41 males and 20 females in the control set. The average age is (64.18 ± 3.71) years. There are 13 cases of squamous carcinoma, 42 cases of adenocarcinoma, 4 cases of adenosquamous carcinoma, and 2 cases of mucoepidermoid carcinoma. In the study set, there are 43 males and 18 females. The average age is (64.02 ± 3.57) years from 53 to 75 years. There are 12 cases of squamous carcinoma, 43 cases of adenocarcinoma, 5 cases of adenosquamous carcinoma, and 1 case of mucoepidermoid carcinoma. The contrast of the two sets of patients' age, carcinoma type, and other clinical general information, *p* > 0.05, there is no statistically extensive disparity between the sets, all patients signed informed consent. Informed consent is required for all patients enrolled in the examination. The therapy and testing methods adopted in this examination are all clinically known safe methods. The general information and clinical data collected in this examination will only be used for examination decomposition and will not be used for other purposes. If you have any discomfort during the therapy, please inform your doctor in charge in time to decide on the next therapy plan. The whole therapy and observation period is 4 weeks, please inform the doctor of the change of your condition in time, do not use any other drugs and other therapy methods for the ailment during the therapy, please inform the doctor if using.

The article "Observation of the Curative Effect of Acupuncture for Tonifying Kidney and Removing Blood Stasis Combined with Radiofrequency Surgery in Patients with NSCLC and the Diagnostic Efficacy of Combined Detection of NTx, BGP, and CYFRA21-1 in the Occurrence of Bone Metastases" was retracted in 2023. Reasons: signs of a paper mill; suspected computer-generated content; unreliable results or conclusions; lack of ethics approval or compliance.

There are five inclusion criteria which include the following: (1) confirmed by histological and cytological diagnosis of NSCLC; (2) expected survival >3 months; (3) KPS scores ranged from 50 to 70; (4) serious ailments of the heart, lung, liver, kidney, and blood system; and (5) signed informed consent

There are eight exclusion criteria which include the following: (1) complicated with other malignant tumors; (2) severe abnormalities of the liver, kidney, and heart function; (3) infectious ailments; (4) people with mental illness; (5) incomplete data, unable to determine the curative effect; (6) poor compliance and inability to cooperate; (7) allergic constitution; and (8) there are patients with local skin ulceration that cannot be treated by acupuncture and point injection.

### 3.2. The Proposed Treatment Method

#### 3.2.1. Control Set

The patients in this set are treated with CT-guided percutaneous radiofrequency ablation, with the main methods as follows: the radiofrequency ablation tumor therapy system (manufacturer: RITAR, MODEL: TM) is adopted. Preoperative CT scan of the tumor is performed, and its longitudinal and transverse diameters are measured to determine the puncture point, depth, and direction of needle insertion. Then, local anesthesia is performed on the puncture point, pleura, and chest wall using 2% lidocaine for routine disinfection towels. Under the guidance of CT, multipole radiofrequency tumor ablation electrode needle is used to puncture the distal edge of the tumor according to the predetermined insertion direction and depth, and CT is used to observe whether the tip reached the predetermined site. After the completion of the puncture, radiofrequency ablation is connected to perform thermal coagulation of the tumor. The ablation temperature is set at 90°C and the time for each target is 15–20 min. Multiple radiofrequency ablation should be performed when the tumor diameter is ≥ 5 cm. After radiofrequency ablation of the tumor, electrocoagulation is used to puncture the needle channel during the withdrawal of the needle to avoid tumor implantation metastasis. After the operation, plain CT scan should be performed on the patient to observe whether there are complications. If there are related complications, corresponding symptomatic therapy should be given to the patient.

The article "Observation of the Curative Effect of Acupuncture for Tonifying Kidney and Removing Blood Stasis Combined with Radiofrequency Surgery in Patients with NSCLC and the Diagnostic Efficacy of Combined Detection of NTx, BGP, and CYFRA21-1 in the Occurrence of Bone Metastases" was retracted in 2023. Reasons: signs of a paper mill; suspected computer-generated content; unreliable results or conclusions; lack of ethics approval or compliance.

#### 3.2.2. Study Set

On the basis of the therapy in the control set, patients in this set are given the combined therapy of kidney tonifying and stasis-removing acupuncture, and the main operation methods are as follows: acupoints are zusanli, Xuanzhong, Dazhu, blood sea, Taixi, Aishi, Houxi, Ququan, Xinyu, and Shuangfei Shu. After routine disinfection of the skin at acupoints with alcohol, disposable sterile acupuncture needles of 0.35 mm × 60 mm are used to adjust the patient's breathing, and the needles are inserted vertically as the patient exhaled. After the gas is obtained, the needle is inserted and gently lifted repeatedly, and finally penetrated into the skin for 30∼50 mm. The patient is given moderate stimulation by the method of smoothing and reinforcing and purging, which made the patient feel acid distension, and the needle is left for 25∼30 min after the needle feeling, during which the needle is used once every 10∼15 min. Both sets are evaluated after 4 weeks of the therapy.

#### 3.2.3. Blood Test

In the morning, 5 ml elbow venous blood is taken from all participants on an empty stomach and centrifuged at 3500 r/min for 10 min with a centrifugation radius of 10 cm. The serum is taken for testing. Serum Pyridinoline cross-linked N-telopeptides of Type 1 collagen (NTx) and bone gla protein are detected by ELISA and Cytokeratin(CyFRA21-1) (kit purchased from Ostex International).

### 3.3. Observation Indicators

#### 3.3.1. Efficacy Evaluation

Refer to clinical Oncology Internal Remedy Manual [20] for evaluation, complete remission (CR): complete absence of pain; extensive relief (PR): extensive relief of pain, normal sleep, and life; mild relief (MR): the pain is less than before the therapy, but there is still extensive pain and sleep disturbance; and ineffective (NR): no relief of pain after the therapy. The total effective rate = (CR + PR) cases/total cases × 100%.

#### 3.3.2. Observation Indicators

The observation index includes the following steps:

1. Compare the quality of life and pain degree of the two sets before and after the therapy: evaluate the quality of life of the patients before and after the therapy according to the KPS score [21], 0∼100 points. A higher score means a better quality of life; NRS [22] scores are used to record the pain degree of patients, with a full score of 10, NRS of no pain is 0, NRS of mild pain is 1–3, NRS of moderate pain is 4–6, and NRS of severe pain is 7–10. The higher the score is, the more severe the pain degree of patients is.
2. The index standards of NTx, BGP, and CYFRA21-1 are contrast between the two sets.
3. The incidence of adverse reactions is contrast between the two sets; incidence of adverse reactions (%) = number of adverse reactions/total number of people × 100%.
4. Bone metastasis in the two sets is observed during the 6-month follow-up.
5. The standards of NTx, BGP, and CYFRA21-1 in patients with and without bone metastasis are contrast.
6. The predictive value of combined detection of NTx, BGP, and CYFRA21-1 for bone metastasis is analyzed.

The article "Observation of the Curative Effect of Acupuncture for Tonifying Kidney and Removing Blood Stasis Combined with Radiofrequency Surgery in Patients with NSCLC and the Diagnostic Efficacy of Combined Detection of NTx, BGP, and CYFRA21-1 in the Occurrence of Bone Metastases" was retracted in 2023. Reasons: signs of a paper mill; suspected computer-generated content; unreliable results or conclusions; lack of ethics approval or compliance.

### 3.4. Statistical Methods

In this examination, all data, data processing all database entry SPSS 26.0, the bank of China, including measurement data line the normal inspection, representation of (‾*x* + *s*), conform to the normal inspection for *F* between the sets, more repeated measurement using MANOVA decomposition of spherical, between the sets data using independent sample *t*-test, paired sample *T* test is used for intraset data, and Mann–Whitney *U* test is used for nonnormal data. The rate is expressed as % and the test is *χ*^2^. Correlation is analyzed by Pearson. The ROC curve is used to compare diagnostic performance. When *p* < 0.05, the disparity between the data is considered statistically extensive.

## 4. Experimental Results

### 4.1. Contrast of Efficacy between the Two Sets

Table 1 shows the contrast of analgesic efficacy between the two sets. It can be observed from Table 1 that the total effective rate in the study set is 90.16%, which is notoriously higher than 67.21% in the control set, and the disparity is statistically extensive (*p* < 0.05).

### 4.2. Contrast of Pain Degree of Quality of Life between the Two Sets before and after the Therapy

Table 2 shows the contrast of the KPS and NRS scores of quality of life between the two sets before and after the therapy. In Table 2, ^*∗*^indicates that contrast with the set before the therapy, *p* < 0.05, the disparity is statistically extensive. It can be observed from Table 2 that the KPS score is lower and NRS score is higher in 2 sets, and there is no extensive disparity (*p* > 0.05) before the therapy. After the therapy, the KPS score is notoriously increased and the NRS score is notoriously subjoined in both the sets, and the KPS score in the study set is notoriously higher than that in the control set, while the NRS score in the study set is notoriously lower than that in the control set (*p* < 0.05).

### 4.3. Contrast of NTx, BGP, and CYFRA21-1 Standards between the Two Sets

Table 3 shows the contrast of NTx, BGP, and CYFRA21-1 standards between the two sets. In Table 3, ^*∗*^ indicates that contrast with the set before the therapy, *p* < 0.05, the disparity is statistically extensive. It can be observed from Table 3 that there are no extensive disparities in the expression of NTx, BGP, and CyFRA21-1 between the two sets (all *p* > 0.05) before the therapy. After the therapy, the standards of NTx, BGP, and CYFRA21-1 in the two sets are enhanced, and the enhancement effect in the study set is notoriously better than that in the control set (all *p* < 0.05).

The article "Observation of the Curative Effect of Acupuncture for Tonifying Kidney and Removing Blood Stasis Combined with Radiofrequency Surgery in Patients with NSCLC and the Diagnostic Efficacy of Combined Detection of NTx, BGP, and CYFRA21-1 in the Occurrence of Bone Metastases" was retracted in 2023. Reasons: signs of a paper mill; suspected computer-generated content; unreliable results or conclusions; lack of ethics approval or compliance.

### 4.4. Contrast of the Incidence of Adverse Reactions between the Two Sets after the Therapy

Table 4 shows the contrast of the incidence of adverse reactions between the two sets after the therapy. It can be observed from Table 4 that the incidence of adverse reactions in the study set is 13.11%, higher than 8.20 in the control set, but there is no extensive disparity (*p* > 0.05).

### 4.5. Contrast of the Occurrence of Bone Metastases between the Two Sets

Table 5 shows the contrast of the occurrence of bone metastasis between the two sets.  Figure 1 shows the contrast of cumulative occurrence of bone metastases between the two sets. Through the above experimental results, it can be observed that the 6-month follow-up of the two sets showed that the incidence of the bone metastasis in the study set is 14.75%, which is notoriously lower than that in the control set (49.18%), and the disparity is statistically extensive (*p* < 0.05).

### 4.6. Contrast of NTx, BGP, and CYFRA21-1 Standards between Patients with and without Bone Metastases

Table 6 shows the contrast of NTx, BGP, and CYFRA21-1 in patients with and without bone metastases. It can be seen from Table 6 that the standards of NTx, BGP, and CYFRA21-1 in the bone metastasis set are notoriously higher than those in the set without bone metastases, with statistically extensive disparities (all *p* < 0.05).

### 4.7. Predictive Value of Combined NTx, BGP, and CYFRA21-1 Detection for Bone Metastases

Table 7 shows the predictive value of combined NTX, BGP, and CYFRA21-1 detection for bone metastases.  Figure 2 shows the ROC curve of the predictive value of NTx, BGP, and CYFRA21-1 combined detection for bone metastases. It is clearly evident from Table 7 and Figure 2 that the ROC area under the ROC curve for prediction and evaluation of bone metastases by NTx, BGP, and CYFRA21-1 combined detection is 0.957, which have high specificity and sensitivity and is notoriously higher than 0.753, 0.726, and 0.719 under the ROC curve by NTx, BGP, and CyFRA21-1 alone. The decomposition and prediction models of the three detection methods are statistically different (*Z* = 2.235, *p* < 0.05).

The article "Observation of the Curative Effect of Acupuncture for Tonifying Kidney and Removing Blood Stasis Combined with Radiofrequency Surgery in Patients with NSCLC and the Diagnostic Efficacy of Combined Detection of NTx, BGP, and CYFRA21-1 in the Occurrence of Bone Metastases" was retracted in 2023. Reasons: signs of a paper mill; suspected computer-generated content; unreliable results or conclusions; lack of ethics approval or compliance.

## 5. Conclusion

The curative effect observation of acupuncture for tonifying the kidney and removing blood stasis combined with radiofrequency surgery in patients with NSCLC and the diagnostic efficacy of combined detection of NTx, BGP, and CYFRA21-1 for bone metastases are investigated. For the NSCLC patients, the application of the kidney-tonifying and stasis-removing acupuncture therapy combined with radiofrequency surgery can notoriously enhance the clinical therapy effect and enhance the quality of life of patients. It can effectively predict the prognosis of bone metastases and is worthy of clinical application.

## Figures and Tables

**Figure 1:** Contrast of cumulative occurrence of bone metastases between the two sets.

**Figure 2:** ROC curve of the predictive value of NTx, BGP, and CYFRA21-1 combined detection for bone metastases.

**Table 1:** Contrast of analgesic efficacy between the two sets.

Sets	CR	PR	MR	NR	Total effective rate
The study set (*n* = 61)	40	10	5	6	55 (90.16)
The control set (*n* = 61)	15	15	11	20	41 (67.21)
*χ * ^2^					9.580
*p*					0.002

**Table 2:** Contrast of KPS and NRS scores of quality of life between the two sets before and after the therapy.

Sets	KPS score		NRS score	
	Before the therapy	After the therapy	Before the therapy	After the therapy
The study set (*n* = 61)	61.47 ± 10.29	84.35 ± 7.58^*∗*^	7.93 ± 1.02	1.22 ± 0.52^*∗*^
The control set (*n* = 61)	60.09 ± 11.05	73.65 ± 11.53^*∗*^	7.86 ± 1.03	3.62 ± 1.07^*∗*^
*t*	0.714	6.056	0.377	−15.756
*p*	0.477	<0.001	0.707	<0.001

**Table 3:** Contrast of NTx, BGP, and CYFRA21-1 standards between the two sets.

Sets	NTx (nmol/L)		BGP (ng/ml)		NCYFRA21-1 (ng/ml)	
	Before the therapy	After the therapy	Before the therapy	After the therapy	Before the therapy	After the therapy
The study set (*n* = 61)	22.96 ± 3.39	8.78 ± 1.78^*∗*^	12.26 ± 2.18	5.32 ± 0.95^*∗*^	17.03 ± 3.63	7.82 ± 1.02^*∗*^
The control set (*n* = 61)	23.15 ± 3.61	13.93 ± 2.09^*∗*^	12.23 ± 2.29	7.13 ± 1.07^*∗*^	17.36 ± 3.57	10.22 ± 2.06^*∗*^
*t*	−0.300	−14.652	0.074	−15.639	−0.506	−13.027
*p*	0.765	<0.001	0.941	<0.001	0.614	<0.001

**Table 4:** Contrast of the incidence of adverse reactions between the two sets after the therapy.

Sets	Nausea	Vomiting	Itchy skin	Constipation	Total incidence rate
The study set (*n* = 61)	2	1	4	1	8 (13.11)
The control set (*n* = 61)	2	2	0	1	5 (8.20)
*χ* ^2^					0.775
*p*					0.379

**Table 5:** Contrast of the occurrence of bone metastases between the two sets.

Sets	Bone metastases	No bone metastases
The study set (*n* = 61)	9 (14.75)	52 (85.25)
The control set (*n* = 61)	30 (49.18)	31 (50.82)
*χ* ^2^	16.621	
*P*	<0.001	

The article "Observation of the Curative Effect of Acupuncture for Tonifying Kidney and Removing Blood Stasis Combined with Radiofrequency Surgery in Patients with NSCLC and the Diagnostic Efficacy of Combined Detection of NTx, BGP, and CYFRA21-1 in the Occurrence of Bone Metastases" was retracted in 2023. Reasons: signs of a paper mill; suspected computer-generated content; unreliable results or conclusions; lack of ethics approval or compliance.

**Table 6:** Contrast of NTx, BGP, and CYFRA21-1 in patients with and without bone metastases.

Sets	NTx (nmol/L)	BGP (ng/ml)	NCYFRA21-1 (ng/ml)
The set without bone metastases (*n* = 83)	6.21 ± 1.17	4.26 ± 0.75	5.26 ± 0.87
The bone metastasis set (*n* = 39)	18.26 ± 2.15	8.97 ± 1.24	13.56 ± 2.72
*t*	−40.072	−25.922	−25.280
*p*	<0.001	<0.001	<0.001

**Table 7:** Predictive value of combined NTX, BGP, and CYFRA21-1 detection for bone metastases.

Indicators	Accuracy	Sensitivity	Specificity	AUC
NTx	76.00	77.50	70.26	0.753 (0.554∼0.763)
BGP	71.50	72.00	75.00	0.726 (0.596∼0.793)
CYFRA21-1	71.00	70.00	76.60	0.719 (0.562∼0.776)
Joint detection	97.00	97.50	94.20	0.957 (0.913∼0.969)

## Data Availability

The simulation experiment data used to support the findings of this study are available from the corresponding author upon request.
